This article has been retracted.

# Homeobox A1 Facilitates Immune Escape and Alleviates Oxidative Stress in Lung Adenocarcinoma

**DOI:** 10.1155/2022/4102666

**Published:** 2022-05-19

**Authors:** Fen Zhao, Hui Tian, Xinchao Liu, Yuanxiazi Guan, Ying Zhu, Peng Ren, Jianbo Zhang, Yinjun Dong, Lei Fu

**Affiliations:** ^1^Department of Radiation Oncology, Shandong Cancer Hospital and Institute, Shandong First Medical University and Shandong Academy of Medical Sciences, Jinan, 250117 Shandong, China; ^2^Department of Radiation Oncology, Shandong Cancer Hospital and Institute, Shandong University, Jinan, 250117 Shandong, China; ^3^Department of Radiation Oncology, Qilu Hospital of Shandong University, Jinan, 250012 Shandong, China; ^4^Cheeloo College of Medicine, Shandong University, Jinan, 250012 Shandong, China; ^5^Affiliated Hospital of Heze Medical College, Heze, 274008 Shandong, China; ^6^Departments of Pathology, Shandong Cancer Hospital and Institute, Shandong First Medical University and Shandong Academy of Medical Sciences, Jinan, 250117 Shandong, China; ^7^Department of Thoracic surgery, Shandong Cancer Hospital and Institute, Shandong First Medical University and Shandong Academy of Medical Sciences, Jinan, 250117 Shandong, China

## Abstract

**Objective:**

Recent studies have demonstrated that homeobox A1 (HOXA1) is upregulated in lung cancer due to RNA modifications (N^6^-methyladenosine), but the specific function of HOXA1 in lung adenocarcinoma (LUAD) remains indistinct. Herein, we investigated the role of HOXA1 in LUAD biology.

**Methods:**

This study presented pancancer analysis of associations of HOXA1 with prognosis, TMB, and immune checkpoints. The expression of HOXA1 was detected in LUAD and normal tissues with immunohistochemistry and western blot. Through least absolute shrinkage and selection operator (LASSO) analysis, HOXA1-derived gene model was conducted in LUAD. Correlations of HOXA1 with immune cell infiltrations, immune checkpoints, HLAs, and chemotherapeutic sensitivity were evaluated. Colony formation, proliferation, and migration of LUAD cells with si-HOXA1 transfection were investigated, and the effects of HOXA1 on T cell exhaustion were assessed *in vitro*.

**Results:**

HOXA1 expression was a risk factor of overall survival, disease-specific survival, and progression-free interval of LUAD. HOXA1 exhibited prominent associations with immune cell infiltration, immune checkpoints, and HLAs. HOXA1-derived gene signature reliably and independently predicted LUAD outcomes. Also, high-risk cases presented increased sensitivity to cisplatin, paclitaxel, docetaxel, vinorelbine, and etoposide. HOXA1 knockdown exhibited an inhibitory effect on proliferation and migration abilities of LUAD cells. Silencing HOXA1 weakened the expression of antioxidative stress markers Nrf2/HO-1 and T cell exhaustion marker CD155 in LUAD cells. Moreover, LUAD cells with HOXA1 knockdown enhanced the CD8+ T cell response.

**Conclusion:**

Our data support the oncogenic function and prognostic significance of HOXA1 that facilitates immune escape and alleviates oxidative stress of LUAD.

## 1. Introduction

Lung cancer represents the major reason for cancer-related deaths, histologically categorized into two main subtypes: small-cell lung carcinoma (SCLC; 15%) [1] and non-small-cell lung carcinoma (NSCLC; 85%) [2, 3]. Lung adenocarcinoma (LUAD) remains the dominating subtype of NSCLC among smokers [4]. This malignancy accounts for most cancer deaths related to smoking, with high risk of metastasis and invasiveness [5]. Nevertheless, the incidence is an increasing trend among young women and never smokers [6]. As estimated, the five-year survival rate remains 19% [7]. Notably, the mechanisms underlying LUAD remain mostly unclear [8]. Hence, there is an urgent need to deeply study the molecular pathogenesis of LUAD to develop more effective therapeutic interventions and reduce mortality. In the past few years, major breakthroughs in the field of cancer immunotherapeutic strategies with immune checkpoint inhibitors (ICIs) have brought a therapeutic revolution for LUAD [9]. Although only a minority of patients present a desirable response to this therapeutic intervention [10], it is urgently required for evaluation of the mechanisms that modulate the tumor immune microenvironment during immunotherapy [11–13].

Homeobox A1 (HOXA1) is a member of homeodomain containing transcription factor family [14–16]. Accumulated evidence suggests that HOXA1 has an oncogenic role in diverse cancer types, including LUAD [14–16]. For instance, evidence suggests that HOXA1 expression is markedly upregulated and possess a moderate diagnostic potential in NSCLC [17]. HOXA1 exhibits prominent high expression in gefitinib-resistant than gefitinib-sensitive NSCLC tissues [18]. HOXA1 upregulation is linked to unfavorable survival outcomes of LUAD patients [19]. Despite this, the mechanisms underlying HOXA1 in LUAD remain unclear. Moreover, HOXA1 may modulate the antitumor immune response through immunosuppression of myeloid-derived suppressor cells (MDSCs) [20]. Lung displays a highly oxidative environment that is tolerated via engaging strictly controlled stress response signaling [21]. Limited evidence shows that oxidative stress can upregulate HOXA1 expression human embryonic stem cells, indicating that HOXA1 might participate in mediating oxidative stress process [22]. Nrf2 is a key stress response mediator [23], and abnormal Nrf2 signaling has been found in 23% of LUAD, demonstrating that Nrf2 dysfunction is the main cancer driver [24]. Suppression of Nrf2 enables to elicit an immunostimulatory tumor microenvironment of lung cancer [25]. Altogether, more investigations should be presented for the prognostic and immunological functions of HOXA1 in LUAD. Herein, the present study was aimed at revealing the function, regulatory mechanisms, and biological significance of HOXA1 in LUAD and at evaluating the clinical significance of HOXA1.

## 2. Materials and Methods

### 2.1. Acquisition of Transcriptome Data

RNA sequencing profiling of 502 LUAD patients was acquired from The Cancer Genome Atlas (TCGA) through the Genomic Data Commons (https://portal.gdc.cancer.gov/). Meanwhile, the matched clinical information was retrieved. Fragments per kilobase per million (FPKM) values were converted to transcripts per kilobase million (TPM) values that were more comparable between samples.

### 2.2. Pancancer Analysis

HOXA1 expression was analyzed in paired tumor and normal specimens across pancancer utilizing the Tumor Immune Estimation Resource (TIMER) 2.0 web server (http://timer.cistrome.org/) [26]. The Spearman correlation analysis was conducted for evaluating the correlations of HOXA1 with tumor mutation burden (TMB) across pancancer. The immune checkpoint gene sets were curated from a previous study [27]. The associations of HOXA1 with immune checkpoints were assessed in each cancer type at the mRNA levels. The univariate Cox regression models were conducted to estimate whether HOXA1 expression was linked to overall survival (OS), disease-survival survival (DSS), and progression-free interval (PFI) for each cancer type.

### 2.3. Identification of HOXA1-Related Genes and Functional Enrichment Analysis

Following the median HOXA1 expression, LUAD cases were classified as high or low expression group. Differential expression analysis was carried out between two groups. Genes with ∣fold change (FC) | >1.5 and false discovery rate (FDR) < 0.05 were selected as HOXA1-related genes. Gene Ontology (GO) and Kyoto Encyclopedia of Genes and Genomes (KEGG) enrichment analyses were presented utilizing clusterProfiler package (version 3.10.1) [28].

### 2.4. Construction of a HOXA1-Derived Gene Model

Univariate analysis was conducted for screening prognostic HOXA1-related genes with *p* < 0.05. A least absolute shrinkage and selection operator (LASSO) Cox regression model was then established with glmnet package (version 4.1-3) [29]. Tenfold cross-validation was utilized to determine the optimal value of penalty parameter *λ*. HOXA1-derived risk score was calculated in accordance with the expression values of candidate variables along with corresponding coefficients. Receiver operating characteristic (ROC) curve was assessed for estimating the predictive precision for risk score. Based on the median value, cases were split into high- or low-risk group. The Kaplan-Meier survival analysis was implemented for estimating OS differences between groups.

### 2.5. Establishment of a Prognostic Nomogram

Through uni- and multivariate Cox regression analyses, independent prognostic indicators were screened among LUAD patients. After combining independent prognostic indicators, a nomogram was established utilizing rms package (version 6.2-0). The predictive precision of this nomogram was confirmed through calibration diagrams.

### 2.6. Analysis of Tumor-Infiltrating Immune Cells

Marker genes of tumor-infiltrating immune cells were collected from a previous study [30]. Single sample gene set enrichment analysis (ssGSEA) was applied for quantifying the abundance levels of 28 immune cell types utilizing GSVA package (version 1.14.1) on the basis of the transcriptomic profiles [31]. The enrichment scores were computed to represent the infiltration of immune cells.

### 2.7. Drug Sensitivity Analysis

Sensitivity to common chemotherapeutic drugs was assessed with the Genomics of Drug Sensitivity in Cancer (https://www.cancerrxgene.org/) project [32]. The half-maximal inhibitory concentration (IC50) was quantified with ridge regression analysis through pRRophetic package (version 1.0.0) [33].

### 2.8. Gene Set Enrichment Analysis (GSEA)

KEGG pathways associated with HOXA1-derived risk score were evaluated utilizing GSEA software (version 1.20.0). The “c2.cp.kegg.v7.1.symbols” file acted as the reference gene set.

### 2.9. Clinical Specimens

In total, 5 pairs of LUAD and normal lung tissues were collected from the patients admitted to the Shandong Cancer Hospital and Institute between March 2020 and January 2021. All subjects did not receive radiotherapy or chemotherapy prior to surgery. This study was approved by the Ethical Committee of Shandong Cancer Hospital and Institute, Shandong First Medical University, and Shandong Academy of Medical Sciences (SDTHEC2020003024). Written informed consent was obtained from each participant.

### 2.10. Immunohistochemistry

Formalin-fixed, paraffin-embedded LUAD and adjacent normal tissues were fixed by 10% formalin for 48 h. The tissues were sectioned into 4 *μ*m thickness. Afterwards, the slices were deparaffinized utilizing xylene as well as antigen retrieval. After blockage, the sections were incubated with primary antibody against HOXA1 (1 : 100; ab72591; Abcam, USA), Nrf2 (1 : 100; 16396-1-AP; Proteintech, China), HO-1 (1 : 100; 27282-1-AP; Proteintech, China), and CD155 (1 : 100; ab267389; Abcam, USA) overnight at 4°C, followed by HRP-labeled secondary antibodies (1 : 200; ab97080; Abcam, USA) for 30 min at room temperature. After being stained by hematoxylin, the sections were scanned with a PathScope pathology slide scanner.

### 2.11. Western Blotting

Total proteins were extracted from tissue or cell specimens utilizing RIPA lysis, which were determined with BCA kit. 20 *μ*g proteins was separated via 10% SDS-PAGE and transferred onto PVDF membranes. After being blocked, they were incubated at 4°C for 12 h with primary antibodies against HOXA1 (1 : 1000; ab72591; Abcam, USA), Nrf2 (1 : 1000; 16396-1-AP; Proteintech, China), HO-1 (1 : 1000; 27282-1-AP; Proteintech, China), CD155 (1 : 1000; ab267389; Abcam, USA), and *β*-actin (1 : 5000; ab179467; Abcam, USA), followed by incubation with secondary antibodies (1 : 5000; ab7090 or ab7097; Abcam, USA) at room temperature for 2 h. Protein band was visualized with ECL kit. Protein expression was quantified utilizing ImageJ software, with *β*-actin as the loading control.

### 2.12. Cell Culture and Isolation of CD8+ T Cells

Human LUAD cell lines A549 and NCI-H1299 were obtained from ATCC company. CD8+ T cells were purified utilizing human CD8+ T Cell Isolation Kit (Miltenyi Biotec, Shanghai, China). All cells were maintained in DMEM (Gibco, USA) containing 10% FBS at 37°C in a humidified incubator with 5% CO_2_.

### 2.13. Cell Transfection

Transfection of 100 nM siRNAs against HOXA1 (GenePharma Co., Ltd., Shanghai, China) into A549 or NCI-H1299 cell line was implemented via Lipofectamine® RNAiMAX reagent (Thermo, USA). Following 24 h, HOXA1 expression was evaluated with western blot. The siRNA sequences were as follows: si-HOXA1#1, 5′-CCCAUGGACUCAUAAACAATT-3′, 5′-UUGUUUAUGAGUCCAUGGGTT-3′; si-HOXA1#1, 5′-GCCUUUGGAAGCUCUUGAATT-3′, 5′-UUCAAGAGCUUCCAAAGGCTT-3′.

### 2.14. Colony Formation Assay

A549 and NCI-H1299 cells (1 × 103 cells/well) were seeded onto a 6-well plate. Following culture for 14 days, formed colonies were fixed by 1 ml 4% paraformaldehyde (Sigma, USA) for 15 min as well as 500 *μ*l Giemsa stain (Sigma, USA) for 20 min at room temperature. The colonies were investigated with an inverted light microscope (Olympus, Japan).

### 2.15. 5-Ethynyl-2'-deoxyuridine (EdU) Staining

Fixation of A549 and NCI-H1299 cells was implemented by 4% paraformaldehyde for 15 min, as well as permeability by 0.3% Triton X-100 reagent for 15 min. EdU staining reagent was added onto wells in the dark for 30 min. Afterwards, antifluorescence quencher was added as well as stained cells were investigated with a fluorescence microscope (Olympus, Japan).

### 2.16. Cell Migration Assay

Transwell (Corning, USA) was utilized for assessing cell migration. A549 and NCI-H1299 cells (3 × 10^5^ cells/ml) with 200 *μ*l serum-free DMEM were planted onto the upper chamber. 600 *μ*l DMEM plus 10% FBS was added to the lower chamber. At 48 h, the cells on the lower chamber were stained by 10% Giemsa for 2 h at room temperature. Stained cells were counted with a light microscope (Olympus, Japan).

### 2.17. Immunofluorescence

A549 and NCI-H1299 cells were maintained in culture dishes. Fixation of the cells was implemented with 4% paraformaldehyde for 15 min. Following being washed by PBS plus 0.05% Tween-20, they were permeabilized utilizing 0.3% Triton X-100 for 5 min, along with blockage by 1% BSA for 30 min as well as incubation with HOXA1 (1 : 100; ab72591; Abcam, USA), Nrf2 (1 : 100; 16396-1-AP; Proteintech, China), and HO-1 (1 : 100; 27282-1-AP; Proteintech, China) antibodies at 4°C overnight, followed by Alexa Fluor® 488 (1 : 100; ab150077; Abcam, USA) or Alexa Fluor® 647 (1 : 100; ab15011; Abcam, USA) antibodies. Nucleus was stained with DAPI. Immunofluorescence images were acquired with a confocal microscope (Olympus, Japan).

### 2.18. Cell Coculture System

CD8+ T cells were sorted as well as cocultured with A549 and NCI-H1299 cells in normal culture plates. The cocultured cells were incubated for two days at 37°C in an atmosphere of 5% CO_2_.

### 2.19. Flow Cytometry

CD8+ T cells were stained by PE-conjugated anti-CD8 antibody. Then, A549 and NCI-H1299 cells were stained by V450-conjugated anti-IFN-*γ* antibody. Cocultured cells were assessed with flow cytometry.

### 2.20. Statistical Analyses

Statistical analyses were carried out utilizing Student's *t* test, Wilcoxon test, or ANOVA followed by Tukey's test with R language (version 4.0.1) or GraphPad Prism (version 8.0). Data are expressed as mean ± standard deviation derived from at least three independent assays. Correlation analysis was carried out with the Pearson or Spearman correlation test. *p* < 0.05 indicated statistically significant.

## 3. Results

### 3.1. Expression Pattern and Immunological and Prognostic Significance of HOXA1 across Pancancer

We firstly presented pancancer analysis of HOXA1 gene with TIMER web server. In Figure 1(a), HOXA1 expression was markedly upregulated in CESC, CHOL, ESCA, glioblastoma multiforme (GBM), head and neck squamous cell carcinoma (HNSC), kidney renal papillary cell carcinoma (KIRP), LUAD, lung squamous cell carcinoma (LUSC), prostate adenocarcinoma (PRAD), and stomach adenocarcinoma (STAD) in comparison to normal tissues. Oppositely, HOXA1 expression was markedly reduced in breast cancer (BRCA), colon adenocarcinoma (COAD), kidney chromophobe (KICH), and kidney renal clear cell carcinoma (KIRC) than normal tissues. TMB is an emerging biomarker of immunotherapeutic response [34]. We analyzed the correlations of HOXA1 with TMB across pancancer. In Figure 1(b), we found that HOXA1 exhibited negative correlations to TMB in BLCA, COAD, LIHC, and UCS but had markedly positive correlations to TMB in KIRC, LGG, LUAD, PAAD, and SARC. Moreover, we observed that HOXA1 was positively associated with immune checkpoints in most cancer types (Figure 1(c)). These data indicated the potential immunological role of HOXA1 across pancancer. Prognostic significance of HOXA1 was further explored in each cancer type via univariate Cox regression analysis. As shown in Figure 1(d), HOXA1 acted as a risk factor for OS of ACC, CESC, HNSC, KICH, KIRC, LAML, LGG, LUAD, THCA, THYM, and UVM. Furthermore, we observed the positive correlations of HOXA1 with worse DSS of ACC, CESC, HNSC, KIRC, LGG, LUAD, UCEC, and UVM (Figure 1(e)). Additionally, HOXA1 was linked to more unfavorable PFI of ACC, CESC, HNSC, KIRC, LGG, LUAD, READ, STAD, and UVM. The above data suggested that HOXA1 may contribute to cancer progression (Figure 1(f)).

### 3.2. HOXA1 Upregulation Is a Risk Factor of LUAD Survival Outcomes

In TCGA cohort, we investigated that HOXA1 expression was markedly upregulated in LUAD than normal specimens (Figure 2(a)). The abnormal expression of HOXA1 was further verified in 5 paired LUAD and adjacent normal specimens. Our immunohistochemistry confirmed that HOXA1 expression was markedly upregulated in LUAD than normal specimens (Figure 2(b)). Western blot also confirmed the prominent upregulation of HOXA1 expression in LUAD (Figures 2(c) and 2(d)). With the median HOXA1 expression, LUAD cases were classified as high or low HOXA1 expression groups. As depicted in Figure 2(e), patients with low HOXA1 expression possessed the survival advantage than those with high HOXA1 expression. The above finding confirmed that HOXA1 upregulation served as an emerging risk factor of LUAD survival outcomes.

### 3.3. Analysis of HOXA1-Relevant Genes and Involved Biological Significance

This study identified 790 HOXA1-relevant genes with ∣FC | >1.5 along with *p* < 0.05 (Supplementary Table 1). Among them, 581 genes exhibited significantly high expression, while 209 genes displayed markedly low expression in high HOXA1 expression group (Figures 3(a) and 3(b)). GO and KEGG enrichment analyses were implemented for uncovering potential biological significance. In Figure 3(c), HOXA1-relevant genes mainly participated in mediating biological processes of B cell-mediated immunity, complement activation, humoral immune response-mediated by circulating immunoglobulin, and protein activation cascade. Also, they might be involved in modulating cellular components of collagen-containing extracellular matrix, collagen trimer, external side of plasma membrane, or immunoglobulin complex (Figure 3(d)). In Figure 3(e), they possessed the molecular functions of antigen binding, extracellular matrix structural constituent, glycosaminoglycan binding, or immunoglobulin binding. Moreover, we investigated that these HOXA1-relevant genes were markedly enriched in cell cycle, chemokine signaling pathway, ECM-receptor interaction, protein digestion and absorption, and viral protein interaction with cytokine and cytokine receptor pathways (Figure 3(f)). The above data highlighted the important biological significance of the HOXA1-relevant genes.

### 3.4. Construction of a Reliable HOXA1-Derived Gene Signature for LUAD Prognosis

The univariate Cox regression analyses uncovered that 358 HOXA1-derived genes were in relation to LUAD prognosis (Supplementary Table2). Afterwards, we presented LASSO Cox regression for selecting highly variable variables. As a result, eight HOXA1-derived genes were included in this model (Figures 4(a) and 4(b)). The HOXA1-derived risk score of each LUAD patient was calculated in line with the following formula: risk score = 0.0728251240226131∗LDLRAD3 expression + 0.0828073308429417∗C1QTNF6 expression + 0.0140814604116393∗ANLN expression + (−0.00119766324400233)∗CRNDE expression + 0.0050720950545627∗LYPD3 expression + 0.0157526948322403∗PKP2 expression + 0.0117856548667349∗IGF2BP1 expression + 0.00659735008359115∗GJB3 expression. ROCs were implemented to estimate the efficacy of this HOXA1-derived gene signature. AUC was >0.6, confirming the favorable predictive performance of this gene signature (Figure 4(c)). With the median risk score, we classified LUAD patients as high or low HOXA1 expression groups (Figure 4(d)). High HOXA1 expression group had more patients with dead status (Figure 4(e)). Heatmap visualized the expression patterns of variables in two groups. We observed the prominent upregulation of CRNDE in low HOXA1 expression group while the marked upregulation of LDLRAD3, C1QTNF6, ANLN, LYPD3, PKP2, IGF2BP1, and GJB3 in high HOXA1 expression group (Figure 4(f)). There was a prominent survival difference in CRNDE between high- and low-risk groups. High-risk patients presented distinctly poorer survival outcomes than low-risk patients (Figure 4(g)). We also evaluated the prognostic value of each variable in LUAD. We observed that ANLN, C1QTNF6, GJB3, IGF2BP1, LDLRAD3, LYPD3, and PKP2 upregulation was positively associated with shortened clinical outcomes across LUAD patients (Figures 4(h)–4(n)). In contrast, low expression of CRNDE was in relation to more unfavorable prognosis of LUAD (Figure 4(o)).

### 3.5. HOXA1-Derived Gene Signature Is an Independent Predictor of LUAD Survival

Through the univariate Cox regression analysis, we investigated that both stage and HOXA1-derived risk score were in relation to worse prognosis of LUAD patients (Figure 5(a)). Moreover, the multivariate Cox regression analysis suggested that both stage and HOXA1-derived risk score may independently predict patients' survival outcomes (Figure 5(b)). Based on the two risk factors, a nomogram was established for LUAD prognosis (Figure 5(c)). Calibration curves confirmed that this nomogram can accurately estimate LUAD patients' one-, three-, and five-year survival duration (Figures 5(d)–5(f)).

### 3.6. Both HOXA1 and HOXA1-Derived Gene Signature Are Associated with Immune Cell Infiltration in the Tumor Microenvironment

By ssGSEA method, we quantified the infiltration levels of diverse immune cells in each LUAD specimen. Compared with low HOXA1 group, we observed the marked increase in infiltration levels of most immune cell types in high HOXA1 expression group (Figure 6(a)). In contrast, eosinophil had the reduced abundance levels in LUAD specimens with HOXA1 high expression. As depicted in Figure 6(b), HOXA1 expression was linked to immune checkpoints and HLA genes across LUAD samples. We also evaluated the difference in tumor immunity between high and low HOXA1-derived risk score. As a result, most immune cell types exhibited markedly increased infiltration levels in high- than low-risk group (Figure 6(c)). However, the decreased abundance of eosinophil was found in high-risk group. Furthermore, we noticed the prominently reduced expression of HLA-DMA, HLA-DRB1, HLA-DQB2, HLA-DRB6, HLA-DRB5, and HLA-DPB1 while the markedly increased expression of HLA-H, HLA-G, HLA-C, HLA-B, HLA-L, and HLA-A in high- than low-risk group (Figure 6(d)). In Figure 6(e), TNFRSF9, CD40, NRP1, CD200, TNFRSF18, HAVCR2, VTCN1, CTLA4, LAIR1, ICOS, TNFSF4, CD274, CD44, PDCD1LG2, CD70, TNFRSF8, VSIR, CD80, TNFRSF4, TNFSF9, PDCD1, IDO1, CD86, CD276, TIGIT, and LAG3 expression displayed marked upregulation in high- than low-risk groups. Meanwhile, IDO2, CD40LG, and TNFSF15 expression was prominently downregulated in high-risk group. Collectively, both HOXA1 and HOXA1-derived gene signatures were linked with tumor immunity of LUAD.

### 3.7. Associations of HOXA1-Derived Gene Signature with Chemosensitivity

We assessed the IC50 value of chemotherapeutic agents in each LUAD specimen. Compared with low-risk group, cisplatin, paclitaxel, docetaxel, vinorelbine, and etoposide displayed lower IC50 values in high-risk group (Figure 7(a)), indicating that HOXA1-derived gene signature could be applied to estimate the responses to cisplatin, paclitaxel, docetaxel, vinorelbine, and etoposide across LUAD patients.

### 3.8. Carcinogenic Pathways Involved in HOXA1

Through GSEA method, we investigated the signaling pathways involved in HOXA1. As depicted in Figure 7(b), HOXA1 upregulation was positively associated with activation of cell cycle, chemokine signaling pathway, cytokine-cytokine receptor interaction, JAK-STAT signaling, pathway in cancer, small cell lung cancer, and Toll-like receptor signaling. This highlighted the tumorigenic effect of HOXA1 in LUAD.

### 3.9. HOXA1 Knockdown Weakens Clone Formation, Proliferation, and Migration of LUAD Cells

To validate the functions of HOXA1 during LUAD progression, HOXA1 expression was silenced by siRNAs against HOXA1 in A549 and NCI-H1299 cells. Western blot confirmed that HOXA1 expression was markedly lowered by si-HOXA1 in A549 and NCI-H1299 cells (Figures 7(c)–7(e)). As depicted in Figures 7(f)–7(h), HOXA1 knockdown weakened clone formation abilities of A549 or NCI-H1299 cell line. Our EdU staining demonstrated that proliferation of LUAD cells was prominently weakened by HOXA1 knockdown (Figures 8(a)–8(c)). Moreover, silencing HOXA1 markedly reduced migration capacity of LUAD cells (Figures 8(d)–8(g)).

### 3.10. HOXA1 Loss Weakens Nrf2/HO-1 Signaling in LUAD Cells

Limited evidence indicates that HOXA1 might participate in mediating oxidative stress [22]. Herein, we detected the expression of antioxidative stress markers Nrf2 and HO-1 in LUAD. Upregulated Nrf2 and HO-1 were found in LUAD than normal specimens (Figures 9(a) and 9(b)). Both in A549 and NCI-H1299 cells, HOXA1 knockdown markedly weakened the expression of Nrf2 and HO-1 (Figures 9(c)–9(i)). This indicated that HOXA1 loss weakened Nrf2/HO-1 signaling in LUAD cells, thereby triggering oxidative stress of LUAD cells.

### 3.11. HOXA1 Modulates T Cell Exhaustion in LUAD

This study further investigated the interaction of HOXA1 with immune cell infiltration in the tumor microenvironment. We evaluated the expression of T cell exhaustion marker CD155. In Figure 10(a), higher CD155 expression was found in LUAD than normal specimens. Intriguingly, HOXA1 silencing markedly reduced CD155 expression in A549 and NCI-H1299 cells (Figures 10(b)–10(d)). A549 and NCI-H1299 cells with HOXA1 knockdown enhanced CD8+ T cell response in the coculture system (Figures 10(e)–10(g)). The above findings demonstrated that HOXA1 may be crucial for modulating CD8+ T cell response through CD155 in LUAD.

## 4. Discussion

ICIs have shown prominent survival benefit in human cancers [35–37]. However, a marked interpatient heterogeneity characterizes immunotherapeutic responses, such as PD-L1 expression and TMB [38]. TMB levels display a prominent association with immune infiltrates in the tumor microenvironment, which can modulate the response to ICIs in LUAD patients [39]. HOXA1 was negatively correlated to TMB in BLCA, COAD, LIHC, and UCS but was positively correlated to TMB in KIRC, LGG, LUAD, PAAD, and SARC. Moreover, HOXA1 displayed positive associations with immune checkpoints in most cancer types. Thus, HOXA1 was in relation to tumor immune response. Our survival analysis demonstrated that HOXA1 was a risk factor of OS, recurrence, and progression in diverse cancer types, including LUAD.

Particularly, our data confirmed the prominent upregulation of HOXA1 expression in LUAD than normal tissues, consistent with previous evidence [40]. HOXA1, a highly conserved homolog in humans, exerts critical roles in cell development and organ formation [41–43]. We identified coexpressed genes of HOXA1 across LUAD samples. Functional enrichment analyses uncovered the regulatory roles of these genes in immunity and inflammation. With LASSO method, we conducted a HOXA1-derived gene signature (containing LDLRAD3, C1QTNF6, ANLN, LYPD3, PKP2, IGF2BP1, GJB3, and CRNDE) for prediction of LUAD prognosis. Following investigations, HOXA1-derived gene signature may reliably and independently predict LUAD survival outcomes. HOXA1-derived gene signature could predict the responses to cisplatin, paclitaxel, docetaxel, vinorelbine, and etoposide across LUAD patients. Combining HOXA1-derived gene signature with stage, we constructed a prognostic nomogram that accurately predicted patients' prognosis. LDLRAD3, C1QTNF6, ANLN, LYPD3, PKP2, IGF2BP1, and GJB3 were risk factors of LUAD prognosis, while CRNDE acted as a protective factor of LUAD outcomes. Previous evidence demonstrates the tumorigenic function of C1QTNF6 in NSCLC [44]. ANLN overexpression is in relation to LUAD metastasis and unfavorable survival outcomes [45]. LYPD3 contributes to LUAD carcinogenesis as well as undesirable prognosis [46]. PKP2 facilitates cellular proliferation and migration through activating EGFR signaling in LUAD [47]. Moreover, PKP2 acts as an important driver of LUAD radioresistance [48]. IGF2BP1 exerts a promoted effect on LUAD progression [49, 50]. CRNDE participates in resistance to EGFR tyrosine kinase inhibitors for EGFR-mutant lung cancer [51]. The above evidence highlights the carcinogenic implication of these HOXA1-derived genes in LUAD.

We investigated that silencing HOXA1 reduced proliferative and move capacities of LUAD cells. The mechanisms by which HOXA1 affects cancer progression through modulating the tumor microenvironment remain indistinct. Thus, we observed the function of HOXA1 on immune cell infiltration across LUAD. Our results demonstrated that HOXA1 expression was linked with immune checkpoints, HLA genes, diverse immune cells, etc. As a critical marker of CD8+ T cell exhaustion, CD155 expression was prominently reduced by HOXA1 knockdown in LUAD cells. In the coculture system, LUAD cells with HOXA1 knockdown could enhance CD8+ T cell response. HOXA1 in normal CD33+ myeloid cells substantially promotes the differentiation of MDSCs as well as suppressive function [52, 53]. Nrf2/HO-1 upregulation triggers aggressive lung cancer as well as is linked to undesirable outcomes [54]. Consistently, our data demonstrated that Nrf2/HO-1 signaling was activated in LUAD than normal tissues. Suppression of HOXA1 enabled to inactivate Nrf2/HO-1 signaling in LUAD cells, thereby triggering oxidative stress of LUAD cells. Altogether, we speculated that HOXA1 may modulate tumor immunity and oxidative stress, thereby affecting the prognosis of LUAD patients. Hence, HOXA1 might become a potential therapeutic target of LUAD. Despite this, several limitations should be pointed out. Firstly, the prognostic significance of HOXA1 requires to be investigated in a prospective cohort. Moreover, the carcinogenic function and mechanisms of HOXA1 will be further verified *in vivo*.

## 5. Conclusion

Collectively, this study uncovered that HOXA1 acted as a risk factor of OS, recurrence, and progression of LUAD. There were marked correlations of HOXA1 with immune cell infiltrations. HOXA1 knockdown reduced proliferative and move capacities of LUAD cells. Also, silencing HOXA1 in LUAD cells induced oxidative stress and ameliorated T cell exhaustion. Hence, HOXA1 may modulate immune cell infiltration in the tumor microenvironment as well as facilitate immune escape and weaken oxidative stress in LUAD.

## Figures and Tables

**Figure 1:** Pancancer analysis of expression pattern and immunogenic and prognostic significance of HOXA1. (a) Expression patterns of HOXA1 in diverse cancer types and matched normal tissue specimens. (b) Correlation analysis of HOXA1 with TMB across pancancer. (c) Heatmap visualizing the associations of HOXA1 with diverse immune checkpoints in each cancer type. Bottom left meant correlation coefficient and upper right corner meant *p* value. Blue represented negative correlation, while red represented positive correlation. ^∗^*p* < 0.05, ^∗∗^*p* < 0.01, and ^∗∗∗^*p* < 0.001. (d–f) Forest plots showing the associations of HOXA1 expression with OS, DSS, and PFI of different cancer types.

**Figure 2:** HOXA1 upregulation is a risk factor of LUAD prognosis. (a) Box plot showing upregulated HOXA1 expression in LUAD than normal specimens. (b) Validation of the expression of HOXA1 in LUAD and adjacent normal tissues utilizing immunohistochemistry. Bar = 5 *μ*m. Magnification, 200x. (c and d) Validation of the expression of HOXA1 in LUAD and paired normal tissues. (e) Kaplan-Meier survival curves of LUAD patients with high and low HOXA1 expression. Survival differences were estimated with log-rank test. ^∗∗^*p* < 0.01.

**Figure 3:** Analysis of HOXA1-relevant genes and involved biological significance in LUAD. (a and b) Volcano plots and heatmap visualizing HOXA1-relevant genes in LUAD. Red meant upregulation while blue or green meant downregulation in LUAD samples with high HOXA1 expression. (c–f) Analysis of biological process, cellular component, molecular function, and KEGG pathways involving HOXA1-relevant genes.

**Figure 4:** Construction of a reliable HOXA1-derived gene signature for LUAD prognosis. (a) Partial likelihood deviance for LASSO coefficient profiling. The red dot indicated the partial likelihood value, the gray line indicated the standard error, and vertical dotted line meant the optimal values by 1 - standard error. (b) LASSO coefficient profiling of candidate genes. (c) ROC curves verifying the predictive accuracy and sensitivity of HOXA1-derived risk score in LUAD survival. (d–f) Distribution of risk score, survival status, and expression pattern of each variable in high or low-risk groups. Vertical dotted line meant the cutoff value of two groups. Red dot represented dead status and green dot represented alive status. Red meant upregulation while green meant downregulation. (g) Kaplan-Meier curves showing survival difference between high and low-risk groups. (h–o) Kaplan-Meier survival curves demonstrating the prognostic value of ANLN, C1QTNF6, GJB3, IGF2BP1, LDLRAD3, LYPD3, PKP2, and CRNDE across LUAD patients.

**Figure 5:** HOXA1-derived gene signature acts as an independent prognostic predictor of LUAD. (a and b) Uni- and multivariate Cox regression analyses for evaluating the associations of clinicopathological features and HOXA1-derived risk score with LUAD prognosis. (c) Establishment of a nomogram in predicting one-, three-, and five-year survival duration. (d–f) Calibration curves verifying the relationships of nomogram-estimated with actual survival duration.

**Figure 6:** Both HOXA1 and HOXA1-derived gene signature are associated with tumor immunity in LUAD. (a) Heatmap showing diverse immune cell infiltrations in LUAD specimens with high or low HOXA1 expression. Blue meant low infiltration levels while red meant high infiltration levels. (b) Correlations of HOXA1 with immune checkpoints and HLA gene family across LUAD samples. Solid line represented a positive correlation and dashed line represented a negative correlation. The darker the box filled, the stronger the correlation. (c) Box plots showing the differences in infiltration levels of diverse immune cells in high and low HOXA1-derived risk score. (d) Box plots demonstrating the differences in mRNA expression of HLA genes in high and low HOXA1-derived risk score. (e) Box plots visualizing the differences in immune checkpoint expressions in high or low HOXA1-derived risk score. ^∗^*p* < 0.05, ^∗∗^*p* < 0.01, and ^∗∗∗^*p* < 0.001.

**Figure 7:** Analysis of chemosensitivity, signaling pathways, and clone formation for HOXA1 in LUAD. (a) Box plots showing the differences in IC50 values of cisplatin, paclitaxel, docetaxel, vinorelbine, and etoposide between high- and low-risk groups. (b) GSEA for identifying signaling pathways involved in HOXA1. (c–e) Western blot showing the expression of HOXA1 in LUAD cells when transfected with si-HOXA1. (f–h) Clone formation of LUAD cells with si-HOXA1 transfection. ^∗∗∗∗^*p* < 0.0001.

**Figure 8:** Silencing HOXA1 reduces proliferation and migration of LUAD cells. (a–c) EdU staining for evaluating the proliferation of A549 and NCI-H1299 cells transfected with si-HOXA1. Bar = 5*μ*m. Magnification, 200x. (d–g) Transwell showing the migration of A549 and NCI-H1299 cells following transfection with si-HOXA1. Bar = 5 *μ*m. Magnification, 200x. ^∗∗^*p* < 0.01, ^∗∗∗^*p* < 0.001, and ^∗∗∗∗^*p* < 0.0001.

**Figure 9:** HOXA1 knockdown weakens Nrf2/HO-1 signaling in LUAD cells. (a and b) Immunohistochemistry showing the expression of Nrf2 and HO-1 in LUAD and normal tissues. Bar = 5 *μ*m. Magnification, 200x. (c–g) Western blot quantifying the expression of Nrf2 and HO-1 in A549 and NCI-H1299 cells transfected with si-HOXA1. (h) Immunofluorescence for the expression of HOXA1 and Nrf2 in LUAD cells following transfection with si-HOXA1. (i) Immunofluorescence for the expression of HOXA1 and HO-1 in LUAD cells under transfection with si-HOXA1. Bar = 5 *μ*m. Magnification, 200x. ^∗∗∗∗^*p* < 0.0001.

**Figure 10:** HOXA1 knockdown enhances CD8+ T cell response through suppressing CD155 expression in LUAD. (a) Immunohistochemistry showing the expression of CD155 in LUAD and normal tissues. Bar = 5 *μ*m. Magnification, 200x. (b–d) Western blot detecting CD155 expression in LUAD cells with si-HOXA1 transfection. (e–g) Flow cytometry measuring IFN-*γ* production in CD8+ T cells after coincubation with LUAD cells transfected with si-HOXA1. ^∗∗∗∗^*p* < 0.0001.

## Data Availability

The data used to support the findings of this study are included within the supplementary information files.

## Abbreviations

SCLC: Small-cell lung carcinoma
NSCLC: Non-small-cell lung carcinoma
LUAD: Lung adenocarcinoma
ICIs: Immune checkpoint inhibitors
HOXA1: Homeobox A1
TCGA: The Cancer Genome Atlas
TIMER: Tumor Immune Estimation Resource
TMB: Tumor mutation burden
OS: Overall survival
DSS: Disease-specific survival
PFI: Progression-free interval
FC: Fold change
FDR: False discovery rate
GO: Gene Ontology
KEGG: Kyoto Encyclopedia of Genes and Genomes
LASSO: Least absolute shrinkage and selection operator
ROC: Receiver operating characteristic
ssGSEA: Single sample gene set enrichment analysis
IC50: Half-maximal inhibitory concentration
GSEA: Gene set enrichment analysis
EdU: 5-Ethynyl-2'-deoxyuridine.

## Supplementary Materials

Supplementary 1 Supplementary Table 1: the information of HOXA1-relevant genes with ∣FC | >1.5 along with *p* < 0.05.

Supplementary 2 Supplementary Table 2: associations of HOXA1-derived genes with LUAD prognosis.
